This article has been retracted.

# Rosiglitazone Alleviates Contrast-Induced Acute Kidney Injury in Rats via the PPAR*γ*/NLRP3 Signaling Pathway

**DOI:** 10.1155/2022/4158692

**Published:** 2022-10-03

**Authors:** Jiayi Wu, Jinhua Huang, En Chen, Xingchun Zheng

**Affiliations:** ^1^Department of Cardiology, Fujian Medical University Union Hospital, Fuzhou, 350001 Fujian, China; ^2^Fujian Heart Medical Center, Fuzhou, 350001 Fujian, China; ^3^Fujian Institute of Coronary Heart Disease, Fuzhou, 350001 Fujian, China; ^4^Fujian Clinical Medical Research Center for Heart and Macrovascular Diseases, Fuzhou, 350001 Fujian, China

## Abstract

**Background:**

This study investigated the effect and mechanism of rosiglitazone on a rat model with contrast-induced acute kidney injury (CI-AKI).

**Materials and Methods:**

The CI-AKI rat model was established from Sprague Dawley rats by furosemide injection (10 ml/kg) to the caudal vein followed by iohexol (11.7 ml/kg). The experimental grouping was randomly allocated into control, model, rosiglitazone, and T0070907 groups. Blood samples were collected from the abdominal aorta. Serum creatinine, urea nitrogen, MDA, and SOD contents were detected by biochemical analysis. TNF-*α* and IL-10 expression was detected by ELISA. Urine creatinine and urine protein were measured following 24-h urine biochemistry testing. Cell pathology and apoptosis were detected by H&E and TUNEL staining, respectively. PPAR*γ*, NLRP3, eNOS, and caspase-3 mRNA expression were detected by qPCR. Caspase-3 and NLRP3 expression were detected by immunohistochemistry.

**Results:**

The CI-AKI rat model was successfully established because the results showed that compared with control, serum creatinine, urea nitrogen, MDA, SOD, TNF-*α*, and IL-10, urine creatinine and urine protein levels were significantly increased in the model group, indicating AKI, but was significantly decreased with rosiglitazone treatment, indicating recovery from injury, while opposite results were obtained with SOD. Apoptosis rate was significantly increased in the model group and significantly decreased with rosiglitazone treatment. NLRP3 and eNOS increased significantly in the model group and decreased significantly with rosiglitazone treatment, while opposite results were obtained with PPAR*γ*. NLRP3 and caspase-3 protein expression was significantly increased in the model group and significantly decreased with rosiglitazone treatment.

**Conclusion:**

Rosiglitazone could alleviate acute renal injury in the CI-AKI rat model by regulating the PPAR*γ*/NLRP3 signaling pathway and should be further investigated as a potential treatment in clinical studies.

## 1. Introduction

In recent years, with the wide application of interventional therapy using multislice spiral computed tomography (CT) and new three-dimensional reconstruction technology, iodine-containing contrast agents are used more frequently and broadly applied in disease diagnosis and treatment. Contrast-induced acute kidney injury (CI-AKI) remains the third most common cause of acute renal insufficiency [1]. The occurrence of CI-AKI seriously affects the rehabilitation of patients and is considered as one of the important complications after interventional therapy, which was reported to be associated with acute hypotension, age, diabetes, dehydration, and others [2–4]. At present, there is still a lack of effective measures to reverse the injury process of CI-AKI. Therefore, understanding the underlying mechanism of CI-AKI and how to effectively alleviate it is of great clinical importance.

The mechanism of CI-AKI remains unclear. At present, it is believed that its occurrence is closely related to contrast agent nephrotoxicity [5, 6]. It includes renal hemodynamic changes, renal tubular toxic injury, inflammatory response, oxidative stress, and apoptosis [7–9]. Destruction of the renal tubular epithelial cell barrier and extensive necrosis of renal tubular epithelial cells are the main pathological features of AKI. Injury and necrosis can also cause a strong host immune response and release of inflammatory factors, including interleukin (IL)-1 and IL-18 [10]. In addition, apoptosis is also responsible for the pathogenesis of AKI [11]. And contrast media can be taken up into the cells and damage mitochondrial function resulting in the increased generation of ROS and cell apoptosis [7]. Therefore, apoptosis is the pathological outcome of most CI-AKI, and inflammatory response and oxidative stress are important ways leading to apoptosis.

Rosiglitazone (RSG) is a synthetic peroxisome proliferator-activated receptor gamma (PPAR*γ*) ligand that activates the PPAR*γ* transcriptional level to regulate downstream target genes [12]. PPAR*γ* is a nuclear receptor involved in immunity and vascular health [13]. Synthetic PPAR*γ* ligand agonists were demonstrated to be renoprotective in diabetic and nondiabetic patients [14].

In this study, a CI-AKI model was established using Sprague Dawley (SD) rats, which were intervened with rosiglitazone and PPAR*γ* inhibitor, to explore whether rosiglitazone can alleviate CI-AKI, its renoprotective functions, and the underlying signaling pathway through which rosiglitazone played its role. We hypothesized that rosiglitazone could alleviate AKI in the CI-AKI rat model by regulating the PPAR*γ*/NLRP3 signaling pathway. The findings of this study might help in the development of a new therapeutic approach for CI-AKI.

## 2. Materials and Methods

### 2.1. Experimental Animals

The experiment was performed in a humane manner in accordance with Ethical Guidelines for Care and Use of Laboratory Animals of Fujian Medical University Union Hospital. This study was approved by the Animal Protocol Committee of Fujian Medical University Union Hospital (2021022301). Twenty-four 250-300 g specific-pathogen-free male SD rats were purchased from Changsha Tianqin Biotechnology Co. Ltd., Changsha, Hunan, P.R. China, with the license no. SCXK (Xiang) 2019-0014. The rats were raised in separate cages and acclimated for 7 days to the laboratory environment (22°C-25°C, 50%-60% humidity, standard 12/12 h light/dark cycle) prior to the experiments.

### 2.2. Laboratory Reagents and Instruments

Dimethyl sulfoxide (DMSO) (D8370), Scott blue buffer (G1865), and eosin (G1100) (Beijing Solarbio Science & Technology Co., Ltd., Beijing., P.R. China); corn oil (8001-30-7), and rosiglitazone (y26M9C56713) (Shanghai Yuanye Bio-Technology Co., Ltd., Shanghai, P.R. China); furosemide (20200902, Ruicheng Weierfu Veterinary Medicine Co., Ltd., Shanxi, P.R. China); iohexol (20100661, Yangtze River Pharmaceutical (Group) Co., Ltd., Jiangsu, P.R. China); PPAR*γ* inhibitor T0070907 (HY-13202/CS-0462, MedChemExpress LLC, NJ, USA); TRIzon reagent (CW0580S), Ultrapure RNA ultra extraction kit (CW0581M), 3,3′-diaminobenzidine (DAB) chromogenic kit (CW0125), and neutral resin (CW01360) (Jiangsu Cowin Biotech Co., Ltd, Jiangsu, P.R. China); HiScript II Q RT SuperMix for quantitative polymerase chain reaction (qPCR) (+gDNA wiper) (R223-01, Vazyme Biotech Co., Ltd., Jiangsu, P.R. China); 2 × SYBR Green PCR Master Mix (A4004M, Xiamen LifeInt Technology Co., Ltd., Xiamen, Fujian, P.R. China); rabbit anticaspase-3 (bs-0081R, 1/100, Bioss Antibodies Inc., Woburn, MA, USA); goat antirabbit IgG (*H* + *L*)-HRP conjugate (ZB-2301, 1/100) and hematoxylin stain (ZLI-9610) (ZSGB-BIO, Beijing, P.R. China); rabbit antinucleotide-binding domain, leucine-rich–containing family, and pyrin domain–containing-3 (NLRP3) (DF7438, 1/100, Affinity Biosciences, Cincinnati, OH, USA); terminal deoxynucleotidyl transferase biotin-dUTP nick end labeling (TUNEL) assay kit (C1088, Beyotime Biotechnology, Shanghai, P.R. China); ultraclear advanced mounting resin (YZB, Baso Diagnostics Inc., Zhuhai, Guangdong, P.R. China); creatinine (Cr) assay kit (C011-2-1), Urine Protein Assay Kit (C035-2-1) (CBB method), and blood urea nitrogen (BUN) ELISA kit (C013-2-1) (Nanjing Jiancheng Bioengineering Institute, Jiangsu, P.R. China); rat IL-10 ELISA kit (MM-0195R2) and rat tumor necrosis factor alpha (TNF-*α*) enzyme-linked immunosorbent assay (ELISA) kit (MM-0180R2) (Jiangsu Meimian Industrial Co., Jiangsu, P.R. China); rat superoxide dismutase (SOD) ELISA kit (SU-B34817) and rat malondialdehyde (MDA) ELISA kit (SU-B30239) (Lun Chang Shuo Biotech, Xiamen, Fujian, P.R. China); UV spectrophotometer (NP80, NanoPhotometer, Munich, Germany); high-speed low-temperature centrifuge (5424R, Eppendorf, Hamburg, Germany); fluorescence PCR instrument (CFX Connect™ Real-Time, Bio-Rad Laboratories (Shanghai) Co., Ltd., Shanghai, P.R. China); automatic sample grinding machine (Tiss-12, Shanghai Jingxin Experimental Technology, Shanghai, P.R. China); auto microplate reader (WD-2102B, Beijing Liuyi Biotechnology Co., Ltd., Beijing, P.R. China); thermal constant temperature incubator (DHP-9054, Biobase Group, Shandong, P.R. China); microscope (BX43), fluorescence microscope (CKX53) (Olympus Corporation, Shinjuku, Tokyo, Japan); and microtome (RM2235, Leica Biosystems, Wetzlar, Germany).

### 2.3. Experimental Grouping and Animal Modeling

1. The experiment was randomly assigned to 4 groups (*n* = 6 rats per group) as follows: (1)control group: no intervention was performed. (2) Model group: a CI-AKI rat model was established by referring to the study of Liu et al. [15]. The rats were deprived of water for 72 h and allowed free access to food [15, 16]. After 72 h, their caudal vein was injected with furosemide (10 ml/kg), followed by iohexol (11.7 ml/kg) 20 min later. Upon completion, free access to food and water was resumed for 24 h. (3) Rosiglitazone group: after successful modeling, 200 mg rosiglitazone hydrochloride powder was accurately weighed and dissolved in 50 ml normal saline. The modeled rats were given intragastric administration of 40 mg/kg rosiglitazone solution per day (divided into three times) for 3 days. Each group was administered at the same time period. Upon completion, free access to food and water was resumed for 24 h. (4) T0070907 group: after successful modeling, 15 mg of PPAR*γ* inhibitor powder (T0070907) was dissolved in 3 ml DMSO solution, and 97 ml of corn oil solution was added and mixed. Each rat was given an intraperitoneal injection of 0.15 mg/ml PPAR*γ* inhibitor T0070907 solution 20 min before intragastric administration of rosiglitazone solution. Upon completion, free access to food and water was resumed for 24 h.

The rats were fed in the metabolic cages after treatment to collect urine samples. Urine Cr and protein (PRO) were determined by 24-h urine biochemistry. 24 h after completing the above procedure, the rats in each group were given an intraperitoneal injection of 45 mg/kg sodium pentobarbital for anesthesia and euthanized. Blood samples were taken from the abdominal aorta of three rats in each group for biochemical analysis of the serum Cr, urea nitrogen, MDA, and SOD contents, and ELISA detection of TNF-*α* and IL-10 levels. The right renal tissue was taken for hematoxylin-eosin (H&E) staining and TUNEL staining for pathological examination and apoptosis detection. The left renal tissue was used for quantitative polymerase chain reaction (qPCR) detection of PPAR*γ*, NLRP3, endothelial nitric oxide synthase (eNOS), and caspase-3 mRNA expression. Caspase-3 and NLRP3 protein expression were detected by immunohistochemistry.

### 2.4. H&E Staining

The renal tissues were collected and rinsed with running water for several hours before dehydration in 70%, 80%, and 90% ethanol solutions, pure alcohol, and xylene (mixed in equal amounts) for 15 min, and xylene I and II for 15 min each (until clear). The tissues were then immersed for 15 min in a mixture of xylene and paraffin (equal amount), followed by 50-60 min each in paraffin I and paraffin II. The tissues were embedded in paraffin and sectioned. The sections were baked, dewaxed, and hydrated, following which they were immersed in distilled water and stained with hematoxylin aqueous solution for 3 min. The sections were then differentiated for 15 s in hydrochloric acid ethanol solution, washed slightly, bluing for 15 s, rinsed with running water, stained with eosin for 3 min, and rinsed with running water gain. Lastly, the sections were dehydrated, cleared, mounted, and examined under a microscope.

### 2.5. ELISA Test

The samples of each group were restored to room temperature. The TNF-*α* and IL-10 levels in the serum samples from the abdominal aorta of rats were determined according to the ELISA kit instructions. The concentrated washing solution and distilled water were diluted by 1 : 20. The standard wells and sample wells were prepared. To each standard well, 50 *μ*l of standards were added at different concentrations. The blank and sample wells were set up. 40 *μ*l of sample diluent was applied to the sample wells of the enzyme-labeled coated plate, followed by 10 *μ*l of samples (final dilution of sample was 5 times), except for the blank wells, and 100 *μ*l of the enzyme-labeled reagent was added to each well. The plate was then sealed with sealing film and incubated for 60 min at 37°C. It was then washed 5 times and patted dry. Chromogenic reagents A and B were added in sequence for 15 min in the dark. Then, 50 *μ*l of stop solution was added to each well to terminate the reaction. The blank wells were adjusted to zero, and each well's absorbance (optical density [OD] value) was measured in sequence under 450 nm wavelength.

### 2.6. Biochemical Testing

The blood and urine samples of each group were restored to room temperature. The contents of serum Cr, urea nitrogen, MDA, and SOD of the abdominal aorta in the rats and the 24-h urine creatinine and PRO were detected according to the biochemical kit instructions. Concentrated washing solution and distilled water were diluted in a 1 : 20 ratio. The following steps of the experiment were the same as in the ELISA test.

### 2.7. TUNEL Detection

The tissue sections were baked for 2 h in an oven at 65°C before being immersed in xylene for 10 min, which was then replaced and left for another 10 min. The sections were placed in 100% (twice), 95%, 80% ethanol, and purified water for 5 min each. Then, this was placed in a wet box, and dropwise Proteinase K working solution (50 ug/ml) was added to each sample and allowed to react at 37°C for 30 min. Then, this was thoroughly washed with phosphate buffer saline (PBS) for 5 min (3 times). The PBS around the tissue was absorbed with absorbent paper. Sufficient amount of TUNEL detection solution was added to each slide and incubated at 45°C for 2 h in the dark. They were then washed with PBS for 5 min (3 times). The liquid on the glass slide was absorbed with absorbent paper; following which antifade mounting media was added and examined under a fluorescence microscope.

### 2.8. qPCR Detection

The renal tissues from each group were grinded into powder. The RNA was extracted, and its concentration and purity were measured with a microultraviolet spectrophotometer. The quality of RNA was determined with agarose gel electrophoresis. A reverse transcription kit was used to synthesize the cDNA, which served as the template. The samples were loaded using the fluorescent dye method, and the program on the fluorescence qPCR instrument was set for the amplification reaction. The PCR reaction conditions were as follows: predenaturation 95°C, 10 min; denaturation 95°C, 10 s; annealing 58°C, 30 s; extension 72°C, 30 s; total 40 cycles. The relative quantitative 2^-△△CT^ method was applied. *β*-Actin was used as the internal reference, and the PPAR*γ*, NLRP3, eNOS, and caspase-3 relative expressions were calculated. All primers were synthesized by Universal Biosystems (Anhui) Co., Ltd., Anhui, P.R. China. PAGE was applied as the purification method. The primer information was as shown in Table 1.

### 2.9. Immunohistochemical Staining

The paraffin sections were deparaffinized in xylene, hydrated with gradient ethanol, and boiled for 3 min in 10 mM citrate buffer (pH 6.0) for antigen retrieval. The sections were treated in 3% H_2_O_2_ for 10 min at room temperature to inactivate the endogenous peroxidase and then, in 5% bovine serum albumin (BSA) for 30 min at 37°C to block nonspecific binding. Subsequently, the sections were incubated at 4°C overnight with the primary antibodies and then for 30 min at 37°C with the corresponding secondary antibody. Color development was performed for 5-10 min using DAB. The degree of staining was measured under a microscope. The sections were counterstained for 3 min with hematoxylin and differentiated in hydrochloric acid and alcohol. After rinsing with water for 1 min, the sections were dehydrated, cleared, mounted, and examined under an optical microscope. The Image-ProPlus 5.0 software was used for analysis.

### 2.10. Statistical Analysis

The SPSS v19 (IBM Corp., Armonk, NY, USA) software was used to analyze the data. The measurement data were expressed as mean ± standard deviation (mean ± SD). Comparisons between multiple groups were performed using a one-way analysis of variance (ANOVA). The Tukey honestly significant difference (HSD) was used for post-hoc test. The experiment was performed 3 times. *P* < 0.05 indicated that the difference was statistically significant.

## 3. Results

### 3.1. H&E Staining of the Rat Renal Tissue

To observe the renal pathological conditions in rats with different treatment (normal renal tissue, CI-AKI, and rosiglitazone treatment), H&E staining was performed to compare the renal tissue sections of each group, where nuclei were shown as blue-purple and cytoplasmic area as red. As shown in Figure 1, the size and shape of the renal tubular lumen of rats in control group were normal, with clear structures, neatly arranged renal tubule epithelial cells, and very few cell necrosis and red blood cell infiltration. But the renal tubules were disordered, the lumina were generally smaller, and most of them were occluded in model group, and the glomerulus was atrophied, renal corpuscle capsule enlarged, renal tubular epithelial cells severely vacuolated and degenerated, cell morphology changed, a large number of red blood cells were seen, and the number of inflammatory cell infiltration in the tubulointerstitium was increased. The interstitial congestion, edema and inflammatory cell infiltration were improved in the rosiglitazone group compared with model group. The T0070907 group showed increased inflammatory cell infiltration and vacuolar degeneration of renal tubular epithelial cells compared with the rosiglitazone group, which was similar to the model group.

### 3.2. ELISA and Biochemistry Analysis of Serum from the Abdominal Aorta and Urine in Rats

As shown in Figure 2, the contents of serum TNF-*α*, IL-10, MDA, SOD, urea nitrogen and Cr of the abdominal aorta, and urine Cr and urine PRO in each group of rats were detected. The contents of serum TNF-*α*, IL-10, MDA, BUN and Cr, and urine Cr and PRO were significantly increased (*P* < 0.05) in the model group compared with the control group, while serum SOD was significantly decreased (*P* < 0.05), indicating that the CI-AKI rat was seriously injured and the CI-AKI model was successfully established. Except for SOD, which was significantly increased (*P* < 0.05), the content of other biomarkers decreased in varying degrees (*P* < 0.05) after rosiglitazone treatment compared with the model group. When rosiglitazone treatment was superimposed with PPAR*γ* inhibitor T0070907, the SOD content decreased significantly, while the other biomarkers increased, indicating that rosiglitazone could effectively improve the renal function and protect against CI-AKI, and the inhibition of PPAR*γ* expression might aggravate the injury of CI-AKI to a certain extent.

### 3.3. TUNEL Detection of Apoptosis in Each Group

Apoptosis is one of the mechanisms of CI-AKI injury. The cell apoptosis of the rat renal tissue was detected using the TUNEL method. As shown in Figure 3, the nuclei showed blue fluorescence, and the apoptotic cells demonstrated green fluorescence. The control and rosiglitazone groups both had few TUNEL-positive cells. The model group had a significantly higher number of TUNEL-positive cells than the control group (*P* < 0.05). When rosiglitazone was superimposed with T0070907, the number of TUNEL-positive cells increased significantly compared with the control group (*P* < 0.05) but decreased significantly compared with the model group (*P* < 0.05), indicating that rosiglitazone treatment could reduce the apoptosis in CI-AKI injury.

### 3.4. The Effect of Rosiglitazone on mRNA Expression in the CI-AKI Renal Tissue

qPCR was performed to detect changes in mRNA expression of PPAR*γ*, NLRP3, eNOS, and caspase-3 in each group.  Figure 4 showed that in the model group, NLRP3, eNOS, and caspase-3 mRNA expression increased significantly (*P* < 0.05, all) compared with the control group, while PPAR*γ* mRNA expression decreased significantly (*P* < 0.05). The NLRP3 and eNOS mRNA expression in the rosiglitazone group decreased significantly (*P* < 0.05, both), PPAR*γ* mRNA expression increased significantly (*P* < 0.05), while caspase-3 mRNA expression showed no significant difference compared with the model group. Rosiglitazone treatment superimposed with PPAR*γ* inhibitor T0070907 showed little difference from the rosiglitazone group, indicating that rosiglitazone has a therapeutic effect on CI-AKI injury to a certain extent, and the mRNA expression levels showed that it had a relatively significant effect on the PPAR*γ*, NLRP3, and eNOS genes.

### 3.5. Effects of Rosiglitazone on Protein Expression of the CI-AKI Renal Tissue

Changes in NLRP3 and caspase-3 protein expression in each group were determined by immunohistochemistry. The blue-purple area indicates the nuclei, and the brown area indicates the target protein expression. As presented in Figure 5, the model group showed significantly increased NLRP3 and caspase-3 protein expression than the control group (*P* < 0.05). After treatment with rosiglitazone, the expression decreased significantly (*P* < 0.05) compared with the model group. It re-increased in the T0070907 group compared with the rosiglitazone group, indicating that from the protein level, the treatment effect of rosiglitazone on CI-AKI injury can be observed.

## 4. Discussion

According to the results of this study, after the CI-AKI rat model was established by iohexol, the arrangement of renal tubules was disordered, the lumen was occluded, the morphology of renal tubular epithelial cells was changed, the tubulointerstitium showed increased cell infiltration, and apoptosis was significantly increased. The model was successfully established. After intervention with rosiglitazone, the interstitial congestion and infiltration were significantly improved, and cell apoptosis was significantly reduced, indicating that rosiglitazone had a certain effect on the treatment of CI-AKI. The strengths of this study were the successful establishment of the CI-AKI (not only assessed by serum creatinine and blood urea nitrogen but also by urine analysis-based studies), potential translational evidence showing that rosiglitazone could have therapeutic effects in such disease, and identifying the underlying mechanism of rosiglitazone in alleviating AKI by regulating the PPAR*γ*/NLRP3 signaling pathway.

By detecting a series of inflammatory factors in the blood and urine of rats, it was found that after modeling, the contents of serum TNF-*α*, IL-10, MDA, SOD, BUN and Cr, and urine Cr and PRO increased significantly. After rosiglitazone intervention, the contents of serum TNF-*α*, IL-10, MDA, SOD, BUN, and Cr decreased significantly, as well as the urine Cr and PRO. Studies have shown that urinary IL-18 in patients undergoing coronary angiography with contrast agents was significantly increased [17]. Previous studies found that contrast media caused an increase in serum urea nitrogen and creatinine[11, 12], tubular necrosis and peritubular capillary congestion [18, 19], MDA [18, 19] and caspase 3 [19], apoptosis [19, 20], and a decreased SOD activity in the kidneys [18, 19], which were concordant with our results.

Conventional studies indicated that the main mechanisms of CI-AKI included local vasoconstriction caused by contrast agents entering the renal vessels and ischemia and hypoxia at the renal cortex and medulla junction. Local oxidative stress and the contrast agent's direct toxic effect on renal tubules eventually result in renal injury, particularly to the renal tubular epithelial cells [21, 22]. Studies have shown that NLRP3 is a cytoplasmic receptor, and researchers have gradually recognized its role in innate immune responses in recent years. Currently, NLRP3 has been recognized as an important inflammatory molecule of pattern recognition receptors [23]. NLRP3 inflammasome, as an important component of innate immunity, plays a critical role in the body's immune response and disease occurrence. Studies have found that inhibiting the NLRP3 inflammasome pathway could reduce renal injury caused by cisplatin [23]. All of the above suggests that the NLRP3 pathway is likely to be activated during acute tubular injury and that NLRP3 inflammasomes may participate in local inflammation during the CI-AKI process. PPAR*γ* is an important member of the nuclear receptor superfamily, participating in inflammatory and immune responses, cell differentiation, proliferation, and apoptosis [9, 24, 25]. After binding to the specific ligands, PPAR*γ* can regulate the transcription of the target genes and inhibit immune cell activation and expression of the inflammatory factors. Caspase-3 is a key executive protease in the apoptosis process and plays the ultimate pivotal role in apoptosis caused by various factors. According to the results, after the SD rats were modeled, the expression of NLRP3 and caspase-3 at the mRNA and protein levels increased significantly, and the expression of PPAR*γ* decreased significantly. After treatment with rosiglitazone, a PPAR*γ* agonist, the NLRP3 and caspase-3 mRNA, and protein expressions decreased, and the expression of PPAR*γ* increased. The expression of eNOS was basically consistent with that of caspase-3. The decrease in apoptosis protein and cell apoptosis rate indicated that NLRP3 was involved in CI-AKI injury, and that rosiglitazone could activate PPAR*γ* to down-regulate the expression of NLRP3, effectively reducing the occurrence of cell apoptosis and achieving a certain therapeutic effect.

This study had several limitations that should be clarified. The effects of different causes of renal injury were not investigated and whether rosiglitazone would be similarly effective in improving the AKI in these different models remained to be determined. Also, only rosiglitazone was used as the main drug, and comparisons with other potential drugs were not performed to assess which would be more effective. Lastly, the upstream and downstream components affecting the PPAR*γ*/NLRP3 pathway were not investigated; thus, further studies are warranted to gain more insight into the mechanism of the nephroprotective action of rosiglitazone.

## 5. Conclusions

The therapeutic mechanism of rosiglitazone on AKI of iodine-containing contrast media may be via upregulating the PPAR*γ* expression and inhibiting the NLRP3 inflammasome signaling pathway. This study initially explored the relationship between rosiglitazone and the PPAR*γ*/NLRP3 signaling pathway and the possible mechanism of action, laying a theoretical foundation for evaluating the role of NLRP3 inflammasome in CI-AKI and performing further in-depth studies on the specific mechanisms.

## Figures and Tables

**Figure 1:** H&E staining of rat renal tissue in each group (400×, scale bar = 100 *μ*m). *n* = 6/group.

**Figure 2:** Changes in the inflammatory factors and renal biomarkers in serum and urine samples in each group. (a) ELISA detection of abdominal aorta blood collection; (b) biochemical analysis of 24 h urine; (c) biochemical analysis of abdominal aorta blood collection. Compared with control group, ^∗^*P* < 0.05; compared with model group, ^#^*P* < 0.05. *n* = 6/group.

**Figure 3:** TUNEL detection of apoptosis in each group (400×, scale bar = 100 *μ*m). Compared with control group, ^∗^*P* < 0.05; compared with model group, ^#^*P* < 0.05. *n* = 6/group.

**Figure 4:** qPCR detection of mRNA expression in renal tissue of each group. Compared with control group, ^∗^*P* < 0.05; compared with model group, ^#^*P* < 0.05. *n* = 6/group.

**Figure 5:** Immunohistochemistry detection of NLRP3 and caspase-3 protein expression in renal tissue of each group (400×, scale bar = 100 *μ*m). Compared with control group, ^∗^*P* < 0.05; compared with model group, ^#^*P* < 0.05. *n* = 6/group.

**Table 1:** The primers used in this study.

Primer name	Primer sequence (5′-3′)	Product length
PPAR-*γ* F	TGCGTCCCCGCCTTATT	114 bp
PPAR-*γ* R	CCTGATGCTTTATCCCCACA	
NLRP3 F	CTCAACAGACGCTACACCCA	99 bp
NLRP3 R	CCACATCTTAGTCCTGCCAAT	
eNOS F	CCACCTGATCCTAACTTGCCT	271 bp
eNOS R	GGAGGTCTTGCACATAGGTCTTA	
Caspase-3 F	TCATGCACATCCTCACTCGT	95 bp
Caspase-3 R	CGGGATCTGTTTCTTTGCAT	
*β*-Actin F	GCCATGTACGTAGCCATCCA	375 bp
*β*-Actin R	GAACCGCTCATTGCCGATAG	

## Data Availability

The data used to support the findings of this study are available from the corresponding author upon request.

## Abbreviations

CI-AKI: Contrast-induced acute kidney injury
CT: Computed tomography
IL: Interleukin
RSG: Rosiglitazone
PPAR*γ*: Peroxisome proliferator-activated receptor gamma
SD: Sprague Dawley
DMSO: Dimethyl sulfoxide
DAB: 3,3′-diaminobenzidine
NLRP3: Nucleotide-binding domain, leucine-rich–containing family, pyrin domain–containing-3
TUNEL: Terminal deoxynucleotidyl transferase biotin-dUTP nick end labeling
Cr: Creatinine
BUN: Blood urea nitrogen
ELISA: Enzyme-linked immunosorbent assay
TNF-*α*: Tumor necrosis factor-alpha
SOD;: Superoxide dismutase
MDA: Malondialdehyde
qPCR: Quantitative polymerase chain reaction
PRO: Protein
HE: Hematoxylin-eosin
eNOS: Endothelial nitric oxide synthase
OD: Optical density
PBS: Phosphate buffer saline
ANOVA: Analysis of variance
HSD: Honestly significant difference.

## References

[1] Nash K., Hafeez A., Hou S. (2002). Hospital-acquired renal insufficiency. *American Journal of Kidney Diseases*.

[2] Brown J. R., Thompson C. A. (2010). Contrast-induced acute kidney injury: the at-risk patient and protective measures. *Current Cardiology Reports*.

[3] Ong M. Y., Koh J. J., Kothan S., Lai C. (2022). The Incidence and Associated Risk Factors of Contrast-Induced Nephropathy after Contrast-Enhanced Computed Tomography in the Emergency Setting: A Systematic Review. *Life*.

[4] Zaki H. A., Bashir K., Iftikhar H., Alhatemi M., Elmoheen A. (2022). Evaluating the Effectiveness of Pretreatment With Intravenous Fluid in Reducing the Risk of Developing Contrast-Induced Nephropathy: A Systematic Review and Meta-Analysis. *Cureus Journal of Medical Science*.

[5] Ramachandran P., Jayakumar D. (2020). Contrast-induced acute kidney injury. *Indian Journal of Critical Care Medicine*.

[6] Lohani S., Rudnick M. R. (2020). Contrast media--different types of contrast media, their history, chemical properties, and relative nephrotoxicity. *Interventional Cardiol ogy Clinics*.

[7] Persson P. B., Hansell P., Liss P. (2005). Pathophysiology of contrast medium-induced nephropathy. *Kidney International*.

[8] Wichmann J. L., Katzberg R. W., Litwin S. E. (2015). Contrast-induced nephropathy. *Circulation*.

[9] McCullough P. A., Choi J. P., Feghali G. A. (2016). Contrast-induced acute kidney injury. *Journal of the American College of Cardiology*.

[10] Tan X., Zheng X., Huang Z., Lin J., Xie C., Lin Y. (2017). Involvement of S100A8/A9-TLR4-NLRP3 Inflammasome pathway in contrast-induced acute kidney injury. *Cellular Physiology and Biochemistry*.

[11] Havasi A., Borkan S. C. (2011). Apoptosis and acute kidney injury. *Kidney International*.

[12] Cuzzocrea S., Pisano B., Dugo L. (2004). Rosiglitazone, a ligand of the peroxisome proliferator-activated receptor-*γ*, reduces acute inflammation. *European Journal of Pharmacology*.

[13] Corrales P., Izquierdo-Lahuerta A., Medina-Gomez G. (2018). Maintenance of Kidney Metabolic Homeostasis by PPAR Gamma. *International Journal Of Molecular Sciences*.

[14] Sarafidis P. A., Bakris G. L. (2006). Protection of the kidney by thiazolidinediones: an assessment from bench to bedside. *Kidney International*.

[15] Liu K., Zhou L. Y., Li D. Y. (2019). A novel rat model of contrast-induced nephropathy based on dehydration. *Journal of Pharmacological Sciences*.

[16] Wu J., Shen J., Wang W. (2022). A novel contrast-induced acute kidney injury mouse model based on low-osmolar contrast medium. *Renal Failure*.

[17] Ling W., Zhaohui N., Ben H. (2008). Urinary IL-18 and NGAL as early predictive biomarkers in contrast-induced nephropathy after coronary angiography. *Nephron Clinical Practice*.

[18] Faubel S., Ljubanovic D., Reznikov L., Somerset H., Dinarello C. A., Edelstein C. L. (2004). Caspase-1-deficient mice are protected against cisplatin-induced apoptosis and acute tubular necrosis. *Kidney International*.

[19] Zhang Y., Yuan F., Cao X. (2014). P2X7 receptor blockade protects against cisplatin-induced nephrotoxicity in mice by decreasing the activities of inflammasome components, oxidative stress and caspase-3. *Toxicology and Applied Pharmacology*.

[20] McCullough P. A. (2008). Contrast-induced acute kidney injury. *Journal of the American College of Cardiology*.

[21] Wong P. C., Li Z., Guo J., Zhang A. (2012). Pathophysiology of contrast-induced nephropathy. *International Journal of Cardiology*.

[22] Maier S., Emmanuilidis K., Entleutner M. (2000). Massive chemokine transcription in acute renal failure due to polymicrobial sepsis. *Shock*.

[23] Kim H. J., Lee D. W., Ravichandran K. (2013). NLRP3 inflammasome knockout mice are protected against ischemic but not cisplatin-induced acute kidney injury. *Journal of Pharmacology and Experimental Therapeutics*.

[24] Wu H., Zhu H., Zhuang Y. (2020). LncRNA ACART protects cardiomyocytes from apoptosis by activating PPAR‐*γ*/Bcl‐2 pathway. *Journal of Cellular and Molecular Medicine*.

[25] Andreucci M., Faga T., Serra R., De Sarro G., Michael A. (2017). Update on the renal toxicity of iodinated contrast drugs used in clinical medicine. *Drug Healthcare and Patient Safety*.

